RETRACTED

# Application of a Remotely Controlled Artificial Intelligence Analgesic Pump Device in Painless Treatment of Children

**DOI:** 10.1155/2022/1013241

**Published:** 2022-04-06

**Authors:** Fengyang Zhang, Shihuan Wu, Meimin Qu, Li Zhou

**Affiliations:** Department of Anesthesiology, Children's Hospital of Nanjing Medical University, Nanjing, Jiangsu 210000, China

## Abstract

In order to effectively improve the application of analgesic pump devices in the treatment of children, a method based on remote control artificial intelligence is proposed. 100 children with dental pulpitis who were treated in a hospital from December 2018 to December 2020 were selected as the research subjects; they were randomly divided into control group and observation group by an equidistant sampling method, with 50 cases in each group. Children in the control group were given articaine and adrenaline anesthesia, and the observation group was treated with articaine and adrenaline combined with a computer-controlled anesthesia system, the anesthesia pain degree and satisfaction degree of the two groups of children were observed and compared. The results showed that the pain score in anesthesia and intraoperative pain score in the observation group was significantly lower than that in the control group, and the differences were statistically significant (*P* < 0.05). The total satisfaction of 96.6% patients in the observation group was significantly higher than that in the control group (84.7%) and the difference was statistically significant (*P* < 0.05). There were no serious complications in both groups. The application of the computer anesthesia system combined with articaine adrenaline in the painless treatment of children's dental pulp proved to have better effects, the treatment compliance is higher, and it is worthy of clinical promotion.

## 1. Introduction

An analgesic pump is a device that continuously pumps fluids and keeps drugs at a steady level in the blood so that fewer drugs can be used for better pain relief. Patients are often allowed to self-press to add an additional infusion dose to the ongoing infusion, so treatment is more individualized, consistent with the large variation in pain sensation. Because the analgesic pump is mainly used for postoperative acute analgesia and maternal labor analgesia, and opioid potent analgesic drugs are often added to analgesic pumps, improper application of the dosage of the drug can often cause life-threatening complications such as respiratory depression in patients; in most domestic hospitals, anesthesiologists are mainly responsible for the preparation and management of analgesic pumps throughout the hospital [1]. When treating children with dental diseases, a preliminary diagnosis of dental disease, related examinations, and a clear diagnosis are required, and then, the treatment plan is clear and implemented. However, due to the influence of related factors, children with dental diseases do not cooperate with clinical diagnosis and treatment operations, which seriously affects the clinical diagnosis and treatment of children with dental diseases. Therefore, when performing clinical diagnosis and treatment of dental patients, limited implementation of treatment for its acute inflammation and pulpitis-related teeth, avoiding the occurrence of pain, building the confidence of the child in diagnosis and treatment, adopting surface anesthesia treatment and injection anesthesia treatment to the children are followed to ensure that the clinical diagnosis and treatment of the children can be successfully completed [2]. The data results in this article show that after comparing the total effective rate of children with dental disease in the experimental group and the reference group, the difference was statistically significant (*P* < 0.05); after comparing the total satisfaction rate of parents of children with dental disease in the experimental group and the reference group, the difference was statistically significant (*P* < 0.05). These statements clarify the advantages of painless operation in the treatment of children's dental diseases. An analgesic pump control method for intelligent infusion is introduced. By setting the sedation depth detection module and/or the respiratory frequency detection module and/or the blood oxygen detection module and the motor drive module, and the processor connected to it to obtain and judge the monitoring signal, the processor evaluates the abnormal signal in time through the judgment of the feedback information of the detection module and automatically adjusts the motor to stop the analgesic pump or slow down the infusion speed in order to reduce the risk of excessive infusion of the analgesic pump. To a certain extent, it reduces the risk of malignancy caused by excessive analgesia with analgesic pumps; however, it still lacks professional anesthesiologists to monitor and manage the abnormal conditions of patients, and safety needs to be paid attention to [3]. In addition, there is no “action” for patients with insufficient analgesia, and it is impossible to achieve individualized analgesia in a true sense.

RETRACTED

However, in reality, due to the large number and scattered distribution of pump patients in the whole hospital, patients have different needs for analgesia in different time periods after surgery; insufficient staffing of the anesthesiology department and cost factors make it impossible for each surgical department to assign a staff member to individualized control and management of the patient's analgesic pump. Continuous pumping at the same speed throughout the entire process is likely to cause severe pain in some patients due to insufficient analgesia, some patients have adverse reactions such as nausea and vomiting, lethargy, urinary retention, numbness of the lower limbs, and itching of the skin due to excessive analgesia, which really affects the patient's analgesic effect and comfort [4]. In addition, the electronically regulated analgesic pumps currently used in clinical practice are often blocked, and the operation is suspended due to mechanical alarms such as insufficient power. The current clinical solution is that the nurse in the ward calls the anesthesiologist, after the anesthesiologist arrives in the ward, the cause of the analgesic pump mechanical alarm is diagnosed and processed, and then the analgesic pump is started. From the patient reporting the alarm problem of the analgesic pump to the nurse calling, to the anesthesiologist arriving in the ward, several hours may pass during this period, and the analgesic pump alarm processing sometimes only needs to be restarted to solve the Wang Y. believes that it is precisely because the anesthesiologist and the patient/family cannot contact in time and provide reliable remote guidance, which undoubtedly increases the time for patients to endure pain and the labor cost for anesthesiologists to manage the analgesic pump [5]. Gao et al. The clinical treatment of dental pulpitis patients mainly adopts pulp opening and pulp extraction treatment plans, but for pediatric patients, controlling the pain during dental treatment and improving the compliance of children with treatment is the key to ensuring the success rate of oral treatment. Compared with traditional lidocaine local anesthesia, oral anesthesia with articaine and epinephrine is more effective, and the incidence of adverse reactions is relatively low, the operation is simple, it has positive significance in improving the compliance of children with treatment [6]. In the work by Yang and Bang, in addition, with the continuous progress and development of medical technology, the computer-controlled local anesthesia system has been applied to the painless treatment of children's teeth and pulp, and has achieved good results; it can ensure painless local anesthesia injection. Computer-assisted systems are used to perform local anesthesia on patients, as it is beneficial to control the injection pressure and injection strength, and can reduce injection pain, make the treatment more comfortable for patients and facilitate the improvement of treatment compliance. This is a new method of anesthesia in recent years, which is conducive to the formation of anesthesia channels, during the injection process. The accuracy of the injection can be ensured, so that a better anesthesia effect can be achieved [7]. The income analysis and research data for this research question are derived from 100 children with dental diseases who attended the hospital and participated in the treatment, 100 children with dental pulpitis who were treated in a hospital from December 2018 to December 2020 were selected as the research subjects, it is randomly divided into a control group and an observation group by means of equidistant sampling, 50 cases in each group. Children in the control group were given articaine and adrenaline anesthesia, the observation group was treated with articaine and adrenaline combined with a computer-controlled anesthesia system, observe and compare the anesthesia pain degree and satisfaction degree of the two groups of children. The results showed that the pain score in anesthesia and intraoperative pain score in the observation group was significantly lower than that in the control group, and the differences were statistically significant (*P* < 0.05). The total satisfaction of 96.6% patients in the observation group was significantly higher than that in the control group (84.7%), and the difference was statistically significant (*P* < 0.05). There were no serious complications in both groups. The aim of this study is to evaluate and study the effect of painless manipulation in the treatment of children with dental diseases. The computer-controlled anesthesia system combined with attevacaine and epinephrine in the treatment of children's dental pulp pain basically achieves painless effect, and is superior to the traditional manual injection of attevacaine, which can better improve the compliance of children's dental pulp and oral treatment, and has better anesthesia effect.

RETRACTED

## 2. Materials and Methods

### 2.1. Composition of an Improved PCA System for Programmed Intermittent Drug Delivery

The improvement of the device is to add a single-chip microcomputer on the basis of the traditional patient-controlled electronic analgesic pump, set the timer on the microcontroller, and connect to the input device and display device of the original electronic analgesic pump. The timer is connected to the PCA pulse control stepper motor through the single-chip microcomputer and achieved an intermittent program control of stepper motors. This design has obtained the “Utility Model Patent Certificate” issued by the State Intellectual Property Office [8].

### 2.2. Pressure Detection of the Infusion System

This experiment uses an Edward pressure sensor connected to an analgesic pump. The entire improved analgesic pump system is connected to the pressure sensor, used to confirm the pressure at the output end during infusion, and recorded the peak pressure of continuous infusion and intermittent infusion; The output is connected to a quantitative beaker to detect the flow at the outflow end. The peak pressure and flow rate were measured 3 times each [9].

### 2.3. Comparison of Peak Pressure between Continuous Dosing and Intermittent Dosing

There was no statistically significant difference in the average value of the peak pressure and flow measurement results between the two groups (*P* > 0.05) (Table 1).

## 3. Simulation Experiment

### 3.1. General Information

100 children with dental pulpitis who were treated in a hospital from December 2018 to December 2020 were selected as the research subjects, and they were divided into two groups, 50 cases in each group, according to whether they used painless operations. Among them, there were 26 males and 24 females in Group A, aged 3–12 years old, with an average of (5.04 ± 0.49) years old. In group B, there were 28 males and 22 females, aged 4–11 years old, with an average of (5.02 ± 0.45) years old. Comparing the general data of the two groups of children with dental diseases, the difference was not statistically significant (*P* > 0.05).

### 3.2. Method

Children with dental disease in the reference group did not use painless operations, after taking tetracaine for topical anesthesia, routinely implement-related diagnosis, and treatment operations. Observation group's dental patients were treated with painless operation and tetracaine was used for topical anesthesia, add bilan anesthesia to the surface anesthesia site for anesthesia treatment, then perform a painless operation, during the injection of the child; it is necessary to pay close attention to the pain and ensure that children can cooperate with them in the implementation of diagnosis and treatment operations [10].

### 3.3. Observation Indicators

(1) To compare and analyze the total effective rate of 100 children with dental disease, effective: the child can keep quiet and cooperate with related operations and can successfully complete the clinical-related diagnosis and treatment of the child, ineffective: the child cried and showed fear for related operations, it is difficult to complete clinical related diagnosis and treatment. (2) To compare and analyze the total satisfaction rate of 100 parents of children with dental diseases, and take a satisfaction survey form, divided into satisfaction and dissatisfaction, satisfaction: The score is 60 points and above, dissatisfied: the score is below 60 points [11].

RETRACTED

### 3.4. Statistical Methods

SPSS21.0 statistical software was used to process the data, and the counting data were expressed as case number (*n*) and percentage (%). *X*^2^ test was adopted, and *P* < 0.05 was considered statistically significant.

## 4. Results and Analysis

### 4.1. Comparison of the Total Effective Rate of the Two Groups

After comparison and analysis of the total effective rate of the two groups of children with dental diseases, the difference was statistically significant (*P* < 0.05). See Figure 1.

### 4.2. Comparison of the Total Satisfaction Rate of the Two Groups

There was a statistically significant difference in the total satisfaction rate of the parents of the two groups of dental children (*P* < 0.05). See Table 2.

### 4.3. Comparison of the Pain Degree of Children before and after Treatment

As shown in Table 3, before treatment, the children's pain degree score has no comparative value, and the difference is not statistically significant (*P* > 0.05); After treatment, the pain degree of group A was higher than that of group B, and the difference was statistically significant (*P* < 0.05) [12].

### 4.4. Analysis

The microcomputer intermittent electronic analgesia pump uses a timer to achieve the purpose of electronically controlled intermittent infusion and manual single administration at the same time. The improved design of the system is relatively simple, as long as a timer is added to the connection of the original analgesic pump automatic control button to realize the selection of the infusion mode. The timer can set two time periods as the choice of dosing interval, in order to meet the needs of clinical application, the method of intermittent drug administration in clinical practice is greatly simplified. Through a meta-analysis of multiple clinical trials, it is believed that continuous intermittent administration can improve patient satisfaction during nerve block and labor analgesia, and reduce total drug consumption. The reason why programmed intermittent injection is more successful than continuous injection is that when a single dose is given, the drug is injected into the epidural space or fascial space and spreads more uniformly [13].

The principle of PCA analgesic pump is realized by discontinuous squeezing silica gel infusion pipe, and liquid entering and releasing are controlled by two vertical rods moving synchronously. A meaningful drive pressure is generated only when the vertical pump, under the action of the motor, squeezes the infusion tube in turn. Our study design examined the pressure of a modified programmed intermittent injection pump. The improved analgesic effect was based on the assumption of increased injection pressure. However, in fact, we detected that the peak pressure of the improved analgesic pump was basically similar to that of the continuous analgesic pump. Therefore, we can conclude that it is not the peak pressure of infusion that influences the infusion outcome, but the infusion and drug metabolism model. Previously, intermittent analgesia was mostly achieved through two analgesic pumps connected to a three-way catheter, one pump for intermittent injection and the other pump for PCA. We connected the timer at the PCA key to realize the parallel path without affecting the PCA key function [14, 15].

RETRACTED

At this stage, due to wrong behaviors in diet, lifestyle, hygiene habits, and tooth use, as a result, there are more and more dental patients, and the incidence of children with dental diseases has also shown a linear upward trend in recent years. After the onset of the disease, children will have symptoms such as bleeding gums, gum inflammation, and swollen gums; if you do not intervene in time, it will cause the children to have loose and missing teeth, which will affect their chewing function and beautiful appearance. Moreover, dental disease can also cause gum inflammation, some inflammatory molecules will flow to various parts of the body along with the blood circulation function of the human body, it affects the body of the child and is not conducive to its healthy development. Therefore, for this kind of disease, children should be given timely and effective treatment to restore the chewing function of children, at the same time, it can also improve the aesthetics of children's teeth, which is conducive to the improvement of the quality of their prognosis. At this stage, early induction and late symptomatic treatment are often used in clinical treatment for children with dental diseases to correct the orientation of the children's teeth, relieve pain and inflammation, and restore the children's tooth growth rate and chewing function. However, in actual operation, because the child is young and has incomplete knowledge of the disease, there is a fear of treatment, which leads to a low degree of cooperation in treatment [16]. Moreover, it is also prone to a variety of abnormal phenomena during treatment, such as crying, resistance, anxiety, etc., which seriously affects normal clinical treatment operations. Moreover, under the influence of this kind of phenomenon, it is easy to cause risk accidents. In order to avoid the occurrence of the above phenomenon and improve the treatment effect, a large number of experimental studies have also been carried out in the clinic, the final result pointed out that the painless treatment of children with dental diseases can not only reduce the pain during the treatment process but also, at the same time, it can also increase the degree of cooperation of the children to ensure that the treatment can be completed smoothly [17].

RETRACTED

The results of this study show that the painless treatment of group B children, the clinical efficacy and satisfaction of family care were higher than that of group A, and the pain degree score was lower than that of group A, and the difference was statistically significant (*P* < 0.05). The results further confirmed the accuracy of relevant medical research, indicating that the painless operation has a positive effect and high application value for children with dental diseases. It can not only reduce the pain performance of children but also have a sedative effect. In combination with the psychological counseling and comfort of doctors and nurses, it can significantly improve its treatment compliance and reduce the treatment risk caused by the psychological stimulation of the child during the treatment process, significantly improving the safety and effectiveness of treatment. Moreover, under the application of painless operation, it can also reduce the worry of the children's family members for the children, it also maintains a good attitude, thereby reducing the occurrence of nurse-patient disputes, and helping to establish a harmonious doctor-patient relationship [18].

During the treatment of pulpitis, operations such as pulp opening and pulp extraction will aggravate the pain of the patient, it makes the patient feel unbearable pain, and the fear in the heart will increase. According to relevant data, among oral medicine patients, about 57% suffer from fear during treatment. Therefore, effective painless techniques must be adopted to ensure the smooth development of treatment. At present, the most common anesthetics in the Department of Endodontics include articaine, lidocaine, proca, and other anesthetics. In addition, the application of computer-controlled anesthesia systems has become more extensive. The application of this system can reduce the pain of anesthesia injection and has a higher clinical application value [19].

Computer-controlled anesthesia system (STA) has been applied to oral clinic in recent years. It is characterized by safety, which can ensure slow and uniform injection, and the flow rate is lower than the patient's pain threshold. At the same time, it can better control the injection strength, grasp the injection site, reduce the pain of injection, and make the patient feel the real comfortable injection. Especially for children with dental diseases, from injection to push medicine basically achieved painless effect. It can be seen from Table 3 that the children's response to pain in the two groups from the beginning of injection to the end of drug push during anesthesia, and the children's response to pain by using attevacaine adrenaline connected to the computer-controlled anesthesia system was lower than that in the control group (*P* < 0.05). In the stage of pulp-out, the children's response to pain is shown in Table 3. The children with attevacaine adrenaline connected to the computer-controlled anesthesia system had significantly lower response to pain than the control group (*P* < 0.05) [20].

RETRACTED

## 5. Conclusion

The computer-controlled anesthesia system combined with articaine adrenaline is basically painless when used in the treatment of dental pulp pain in children, at the same time, it is better than the traditional hand injection method of articaine, which can better improve the compliance of children's dental pulp oral treatment, and the anesthesia effect is better; at the same time, complications such as nerve injury and hematoma are avoided, and the pain of children is less, and the incidence of dental fear in children is reduced. Therefore, the computer-controlled anesthesia system is worthy of promotion.

## Figures and Tables

**Figure 1:** Comparison of the total effective rate of the two groups of children with dental disease.

**Table 1:** Peak pressure and flow test results of two groups of analgesics infusion.

Method	Set value	Peak pressure	Flow

Intermittent dosing	10	26.7 ± 0.4	10
Continuous dosing	10	23.8 ± 0.5	10
Intermittent dosing	5	27.2 ± 0.4	5
Continuous dosing	5	24.2 ± 0.6	5

**Table 2:** Comparison of the total satisfaction rate of the two groups of children with dental diseases.

Grouping	Dissatisfied	Satisfy	Overall satisfaction rate

Group A	13	36	72
Group B	3	47	94
*X* ^2^			8.5755
*P*			0.034

**Table 3:** Comparison of the degree of pain in children after treatment.

Grouping	Number of cases	Before therapy	After treatment

Group A	50	7.02 ± 1.49	5.87 ± 1.16
Group B	50	6.97 ± 1.54	3.31 ± 0.24
*X* ^2^		40.805	37.170
*P*		0.001	0.001

## Data Availability

The data used to support the findings of this study are available from the corresponding author upon request.
